# Bioadhesive hydrogel comprising bilirubin/β-cyclodextrin inclusion complexes promote diabetic wound healing

**DOI:** 10.1080/13880209.2021.1964543

**Published:** 2021-08-23

**Authors:** Qing Yao, Yannan Shi, Xing Xia, Yingying Tang, Xue Jiang, Ya-Wen Zheng, Hailin Zhang, Ruijie Chen, Longfa Kou

**Affiliations:** a Department of Pharmacy, The Second Affiliated Hospital and Yuying Children’s Hospital of Wenzhou Medical University, Wenzhou, China; b School of Pharmaceutical Sciences, Wenzhou Medical University, Wenzhou, China; c Central Laboratory, The First Affiliated Hospital of Wenzhou Medical University, Wenzhou, China; d Department of Children’s Respiration Disease, The Second Affiliated Hospital and Yuying Children’s Hospital of Wenzhou Medical University, Wenzhou, China

**Keywords:** Thiolated polyglutamic acid, bilirubin inclusion complex, rheological characterization, anti-inflammation, macrophage polarization, tissue remodelling

## Abstract

**Context:**

Chronic non-healing diabetic wound therapy is an important clinical challenge. Manipulating the release of bioactive factors from an adhesive hydrogel is an effective approach to repair chronic wounds. As an endogenous antioxidant, bilirubin (BR) has been shown to promote wound healing. Nonetheless, its application is limited by its low water solubility and oxidative degradation.

**Objective:**

This study developed a bilirubin-based formulation for diabetic wound healing.

**Materials and methods:**

Bilirubin was incorporated into β-CD-based inclusion complex (BR/β-CD) which was then loaded into a bioadhesive hydrogel matrix (BR/β-CD/SGP). Scratch wound assays were performed to examine the *in vitro* pro-healing activity of BR/β-CD/SGP (25 μg/mL of BR). Wounds of diabetic or non-diabetic rats were covered with BR or BR/β-CD/SGP hydrogels (1 mg/mL of BR) and changed every day for a period of 7 or 21 days. Histological assays were conducted to evaluate the *in vivo* effect of BR/β-CD/SGP.

**Results:**

Compared to untreated (18.7%) and BR (55.2%) groups, wound closure was more pronounced (65.0%) in BR/β-CD/SGP group. In diabetic rats, the wound length in BR/β-CD/SGP group was smaller throughout the experimental period than untreated groups. Moreover, BR/β-CD/SGP decreased TNF-α levels to 7.7% on day 3, and elevated collagen deposition and VEGF expression to 11.9- and 8.2-fold on day 14. The therapeutic effects of BR/β-CD/SGP were much better than those of the BR group. Similar observations were made in the non-diabetic model.

**Discussion and conclusion:**

BR/β-CD/SGP promotes wound healing and tissue remodelling in both diabetic and non-diabetic rats, indicating an ideal wound-dressing agent.

## Introduction

Diabetes is a prevalent disease globally, characterized by high blood glucose (Lovic et al. 2020), primarily caused by insulin insufficiency. In diabetic patients, the development of diabetic wound is influenced by peripheral neuropathy, vessel damage, hyperglycaemia, and decreased immune function. As such, most diabetic wounds may progress to chronic wound, manifested by delayed healing, causing diabetic limb ulcer, venous haemorrhagic ulcer, gangrene, and amputation (Bowers and Franco 2020). Hyperglycaemia-induced advanced glycation end-products (AGEs) and reactive oxygen species (ROS) in diabetic wounds exert chronic and persistent inflammation cascade reactions (Berezin 2016). The resultant inflammation influences the healing rate of diabetic wound.

Bilirubin (BR), the end product of haem metabolism, plays an antioxidant and anti-inflammatory effect in the body (Yao, Jiang, Kou, et al. 2019). It eliminates ROS, which promotes oxidative stress and inflammation, the two cyclical processes (Yao, Chen, et al. 2020; Yao, Jiang, et al. 2020). Previously, we found that BR promoted islet transplantation in diabetic mice by preventing inflammation (Yao, Jiang, Huang, et al. 2019; Yao, Huang, et al. 2020; Yao, Sun, et al. 2020). Specifically, biliverdin, a superior product of BR, exerts antioxidant and anti-inflammatory effects (Yao, Lan, et al. 2020). Research has confirmed that BR and biliverdin cycle regulate antioxidant systems to promote endothelial cell protection (Jansen et al. 2010). The low water solubility of BR limits its clinical application. Bilirubin has long been considered a metabolic toxin. Plasma levels of bilirubin is elevated in patients with hepatitis or liver failure, and cause hepatic coma, and even death (Vítek 2020). Several strategies have been used to remove bilirubin from the blood using a dialysis system containing adsorbents (Qiao et al. 2020; Wu et al. 2020; Song et al. 2021). β-cyclodextrin (β-CD), a cyclic heptamer of glucose α-1, 4 d-glucopyranoside that creates a toroid structure with a hollow hydrophobic core, was adopted to remove BR from plasma (Inderbitzin et al. 2010; Wang et al. 2012; Liu et al. 2017). These studies also demonstrated that BR inclusion complexes can be used to increase the druggability of BR. Inspired by these studies, a β-CD-based BR inclusion was developed in this study to promote wound healing.

Hydrogels formed by hydrophilic polymers possess good biocompatibility, variable structure, flexibility, and can adequately cover wounds caused by surgical trauma (Hu and Xu 2020). Hydrophilic hydrogels provide a humid environment, act as a physical barrier that prevents bacteria invasion, and present a porous network that allow loading of multiple therapeutic agents thereby promoting wound healing. Poloxamer has been widely studied as a suitable hydrogel polymer that accelerate tissue regeneration and wound healing (Yao, Zheng, et al. 2020). Incorporating functional materials into the poloxamer hydrogel system creates a hydrogel system with favourable properties for wound healing (Li et al. 2019). It has been reported that γ-polyglutamic acid (γ-PGA) hydrogel forms a no-fallen shape and adheres to the skin. Thiolation may further enhance the adhesiveness of the hydrogel (Gajendiran et al. 2018; Yang et al. 2020). Previously, we found that thiolated γ-PGA hydrogel improved the biocompatibility and adhesiveness of an ocular hydrogels thereby accelerating cornea repair (Xu et al. 2019). Therefore, we developed a bioadhesive hydrogel using poloxamer and thiolated γ-PGA polymer coupled with β-CD-based BR inclusion for wound healing.

Here, based on the performance of β-CD based absorbents for bilirubin removal, we formulated inclusion complexes of bilirubin using β-cyclodextrin (BR/β-CD) as the drug delivery system. Then BR/β-CD was further modified into a thiolated polyglutamic acid-based bioadhesive hydrogel (BR/β-CD/SGP) to achieve controlled release of BR and accelerate chronic wound healing (Scheme 1). The formation of BR/β-CD inclusion complex and bioadhesive hydrogel were systemically characterized. The BR/β-CD inclusion complex appeared as an orange powder, soluble in aqueous solution, and stable in the presence of light, while retaining its antioxidative and anti-inflammatory properties. The BR/β-CD/SGP hydrogel promoted closure of chronic wounds in streptozotocin (STZ)-induced diabetic mice. These results demonstrated that BR/β-CD/SGP hydrogels can effectively promote diabetic wound healing.

**Scheme 1.** The schematic graph showing the bioadhesive hydrogel containing BR/β-CD inclusion complexes used to promote diabetic wound healing.

## Materials and methods

### Materials

Bilirubin (BR), β-CD, γ-PGA (700 kDa), cysteamine (Cys), 1-ethyl-3-(3-dimethylaminopropyl)-carbodiimide (EDC), *N*-hydroxy-succinimide (NHS), morpholine ethanesulfonic acid (MES), and 3-(4,5-dimethyl thiazol-2-yl)-2,5-diphenyl tetrazolium bromide (MTT) were obtained from Sigma-Aldrich (St. Louis, MO, USA). Poloxamer F127 was obtained from BASF (Ludwigshafen, Germany). DMEM medium, foetal bovine serum (FBS), bovine serum albumin (BSA), and trypsin were purchased from Gibco (Gibco-BRL, Carlsbad, CA, USA). Haematoxylin and eosin (H&E) staining kit, primary antibodies of tumour necrosis factor α (TNF-α) (ab215188), myeloperoxidase (MPO) (ab208670), CD86 (ab243887), vascular endothelial growth factor (VEGF) (ab32152), transforming growth factor β (TGF-β) (ab215715), and fibroblast growth factor 1 (FGF-1) (ab179455) were purchased from Abcam (Shanghai, China).

### Cell culture

HUVEC cells were maintained in a thermostatic incubator with 5% CO_2_ and 37 °C and cultured in Gibco DMEM with 10% FBS and 100 U/mL penicillin/streptomycin.

### Preparation and characterization of BR/β-CD inclusion complex

The BR/β-CD inclusion complex was prepared by solvent evaporation method. First, 100 mg BR was dissolved in 10 mL chloroform, while β-CD was dispersed in 10 mL methanol. Next, the BR solution and β-CD solution were mixed by stirring, and the organic solvents were removed by rotary evaporation. Thereafter, 10 mL distilled water was added to redisperse the samples, sonicated and stirred at 50 °C until it fully dissolved. The samples were purified by recrystallization and lyophilized.

BR/β-CD inclusion complex was characterized by Fourier transform infra-red (FTIR) spectrophotometer (Equinox 55, Bruker, Karlsruhe, Germany), X-ray diffractometer (XRD) (Thermofisher, China), thermogravimetric analysis (TGA) and differential scanning calorimetry (DSC) analyzer (Greifensee, Switzerland) as previously reported (Yao, Lin, et al. 2020). The stability of the drug after being included in the cyclodextrin was evaluated by monitoring changes in drug concentration after exposure to light for 7 days.

### Preparation of BR/β-CD/SGP hydrogel

Thiolated γ-PGA was synthesized and characterized as previously reported (Xu et al. 2019). Briefly, 500 mg PGA was dissolved in the 100 ml MES solution (1 mg/mL, pH = 6.0). Then, 190 mg EDC and 600 mg NHS were added to the solution and stirred for 40 min. Next, 1.2 g Cys was added into the solution which was stirred for 6 h in a darkness. After reaction, the sample was dialyzed for 48 h in a medium containing 0.1 mM H_2_O_2_. Thiolated γ-PGA power was obtained after lyophilization.

Then, 0.5 mg thiolated γ-PGA and 2 g poloxamer were dissolved into the 10 mL distilled water. Subsequently, the solution was kept still overnight to form the SGP hydrogel. Poloxamer hydrogel (P) and γ-PGA based-poloxamer hydrogel (GP) were prepared for comparison. BR/β-CD/SGP hydrogel was prepared by adding BR/β-CD lyophilized powder (BR concentration of 1 mg/mL) into thiolated γ-PGA/poloxamer solution during the hydrogel process. BR/β-CD/SGP hydrogel was stored at 4 °C.

### Characterization of BR/β-CD/SGP hydrogel

First, the hydrogels were immersed in double-distilled water for swelling equilibrium, then freeze-dried. After the samples were sprayed with a thin gold layer, the cross-sectional morphologies of lyophilized samples were visualized under a scanning electron microscope (SEM) (Hitachi SU8020, Japan), and the accelerating voltage was kept at 30 kV.

Enzymatic degradation was performed to evaluate the degradation rate of BR/β-CD/SGP hydrogel in papain (0.05 mg/mL) containing pH 7.4 buffer using a thermostatic oscillator controlled at 37 °C. At each time point, the samples were removed and weighed. The *in vitro* degradation rate was calculated by dividing the dry weight after degradation (W_t_) with the initial dry weight of the gel (W_0_) as follows: relative weight remaining = (W_t_/W_0_) × 100%.

Rheological behaviour was measured using a rheometer (TA-AR-G2) at temperatures ranging from 10 to 40 °C. Storage modulus (G′) and loss modulus (G′′) of hydrogel samples were measured using parallel plates at room temperature in oscillatory mode for 10 min (Gap size = 1 mm, strain = 1.0%).

The adhesive strength of the hydrogel towards host tissue was established using fresh SD rat skin. Briefly, the skin was cut into 10 × 10 mm rectangle and placed in pH 7.4 PBS before use. Exactly 100 µL of BR/β-CD/SGP hydrogel was coated on the skin surface, and another piece of skin was placed onto the hydrogel. For complete adhesion, the porcine skin was kept at room temperature for 2 h. The lap shear test was performed on a Materials Test system (MTS Criterion 43, MTS Criterion) to analyze the adhesion properties of these hydrogels.

### *In vitro* release profile of BR/β-CD/SGP hydrogel

*In vitro* release of BR from BR/β-CD/SGP hydrogel was performed using a modified dialysis method (Yao, Liu, et al. 2019; Yao, Lin, et al 2020; Kou, Sun, Xiao, et al. 2020). Briefly, 20 mL of the BR/β-CD/SGP hydrogel was incubated with PBS (pH 7.4) containing 0.5% sodium dodecyl sulphate and stirred at 37 °C thermostatic oscillator. About 400 μL of the supernatant was collected at different times and a fresh solution was added. The released BR was analyzed through UV-vis spectroscopy. The amount of released BR was normalized to the initial concentrations.

### MTT test

HUVEC was grown in the 96-well plate and incubated with different concentrations of BR or BR/β-CD or BR/β-CD/SGP hydrogel. After 24 h, 10 μL MTT solution (5 mg/mL) was added to each well and incubated at 37 °C for 4 h. Subsequently, the medium was removed and DMSO was added to dissolve formazan. Supernatants from each well were collected and measured at 570 nm by microplate assay (Thermo Fisher, China).

### *In vitro* scratch wound assay

HUVEC was grown in 24-well plates and vertically scraped with the tips of pipette heads. Then, BR or BR/β-CD or BR/β-CD/SGP (25 μg/mL of BR) was added into the 24-well plates and incubated for 24 h. The wound migration was then visualized under an inverted microscope (Thermo Fisher, China).

### Diabetic wound model and drug treatment

All animals were purchased from Shanghai Laboratory Animal Centre (Shanghai, China) and allowed free access to water and food in an appropriate environment with a 12 h light/dark cycle. Animal experiments were performed following the “Guide for the Care and Use of Laboratory Animals” published by the US National Institutes of Health and approved by the Institutional Animal Care and Use Committee of Wenzhou Medical University.

To establish a diabetic rat model, rats were fasted for 12 h before intraperitoneal injection with 150 mg/mL streptozotocin (STZ). The diabetic model was recognized as successful when blood glucose was above 100 mM for 2 weeks. Then, the rats were divided into 3 groups (*n* = 6), i.e., diabetic rats without treatment (DM), diabetic rats with BR (DM + BR), and diabetic rats with BR/β-CD/SGP hydrogel (DM + BR/β-CD/SGP). All the rats were then anaesthetized and depilated to expose the entire back, and a 2 cm diameter circle was cut from a similar position on the back of the rats. This wound model was also created on non-diabetic rats, including two groups, i.e., normal rats without treatment (Nor) and normal rats with BR/β-CD/SGP hydrogel (Nor + BR/β-CD/SGP). BR or BR/β-CD/SGP hydrogel was administered by direct coating on the wounds in equal BR concentrations (1 mg/mL).

### H&E and immunohistochemical staining

Skin tissues on day 3 and day 7 post-administration were fixed with 4% formaldehyde for 48 h, dehydrated via alcohol gradient method, and embedded in paraffin. Then, the tissue samples were further sectioned (5 µm) and stained based on the H&E kit protocols.

Immunohistochemistry was performed as previously reported (Kou et al. 2019; Kou, Sun, Jiang, et al. 2020; Zhao et al. 2020). Endogenous peroxidase was blocked with 3% H_2_O_2_ for 10 min. Antigen retrieval was performed with trypsin for 10 min, and non-specific binding was blocked with 5% BSA for 30 min. Samples were then incubated with blocking buffer diluted primary antibodies overnight at 4 °C, TNF-α (1:200, Abcam), FGF-1 (1:200, Abcam), collagen (1:200, Abcam), VEGF (1:200, Abcam), CD86 (1: 100, Abcam), MPO (1:1000, Abcam). Samples were then incubated with horseradish peroxidase (HRP)-conjugated secondary antibodies diluted in blocking buffer for 1 h. The slides were treated with Diaminobenzidine (DAB) for 2-3 min, and then counterstained with haematoxylin.

### Statistical analysis

Statistical tests were performed using GraphPad Prism 7 software (GraphPad, USA) and SPSS 22.0 software (IBM, USA). Unless otherwise stated, data were shown as the mean ± SD. Comparison between groups was conducted by one-way ANOVA followed by Bonferroni test. *p* < 0.05 was considered statistically significant.

## Results and discussion

### Characterization of BR/β-CD inclusion complex

BR/β-CD inclusion complex was prepared using solvent evaporation method and characterised by FITC, UV, XRD, TGA, DSC, and stability analysis (Figure 1). The FTIR spectra of the BR, β-CD, and BR/β-CD are shown in Figure 1(A). BR exhibited sharp peaks at 3409 and 1698 cm^−1^, belonging to the N–H stretch band in the pyrrole ring and carboxyl in the BR molecular structure. β-CD showed characteristic peaks at 3417 cm^−1^ of -OH stretching vibration and 2909 cm^−1^ of the C–H stretching vibration, and several small absorption peaks of the stretching vibration of the C–O bond in the fingerprint region including 1157, 1081, 1030, and 939 cm^−1^ (Qiu et al. 2014). The results revealed that FT-IR of BR/β-CD and β-CD were highly similar due to the BR incorporated in the complex and the overlapping absorption bands of BR and β-CD. Nevertheless, the most significant absorption rate of pure BR at 1698 and 1200 cm^−1^ occurred in the BR/β-CD inclusion complex, indicating the presence of BR and molecular interaction between BR and β-CD. These results suggest that BR was incorporated into the non-polar cavity of β-CD.

**Figure 1.** Characterization of BR/β-CD (A) FTIR spectra, (B) UV spectra, (C) XRD, (D) TGA, and (E) DSC of BR, β-CD, BR/β-CD, and BR + β-CD (the mixture of BR and β-CD). (F) Bilirubin content of BR and BR/β-CD after standing for 7 days. The recorded appearance images of (G) BR and (H) corresponding UV spectra in 7 days. The recorded appearance images of (I) BR/β-CD and (J) corresponding UV spectra in 7 days. **p < 0.05 compared to the BR solution group.

The formation of an inclusion complex was verified using the ultraviolet spectra (Figure 1(B)). It was found that β-CD showed nearly no absorption activity throughout the tested wavelength, hence, its absorbance was neglected. BR exhibited a strong absorption peak at 450 nm. The inclusion complex of BR and β-CD had a decreased absorption spectrum compared to BR, indicating a successful preparation of BR/β-CD inclusion.

Powder X-ray diffractometry (PXRD) is a powerful method used to detect CD complexation of small compounds in powder or crystalline states. It differentiates the formation of complexes due to clear differences between the diffraction pattern superposition of the components and the diffraction pattern of the inclusion complex. Several sharp diffraction peaks from the XRD pattern of BR indicated the crystalline state (Figure 1(C)). The diffraction peaks of β-CD had a typical cage-type structure (Kayaci and Uyar 2011). The PXRD patterns of the inclusion complex were different from those of β-CD, BR, or physical mixture. The difference between the spectra of β-CD and the inclusion complex was due to the interaction of β-CD with BR. The diffraction peaks of BR were absent from the XRD pattern of BR/β-CD indicating that the inclusion complex had formed a head-to-head channel-type structure (Luo et al. 2012). Specifically, the physical mixture of BR and β-CD showed a simple stack of BR and β-CD in the XRD pattern, significantly different from that of the BR/β-CD inclusion.

TGA-DSC is a technique used to detect the complexation process. The TGA-DSC curve of β-CD was consistent with findings from previous studies (Figure 1(D,E)) (Dos Passos Menezes et al. 2017). The rapid decline in the DSC curve near 330 °C indicated the decomposition of water (Figure 1(E)). A small thermal event that appeared near 310 °C in the DSC analysis of BR reflected a crystalline phase transition, which was under the melting point shown in TGA analysis (Figure 1(D)). In contrast, two endothermic peaks were seen in the DSC curves of BR/β-CD, suggesting successful incorporation of BR into the cavities of the β-CD. TGA results showed that the melting point of BR/β-CD slightly moved to a lower temperature. The reduction in the endothermic peak was explained due to the replication of BR with water in the β-CD cavity when complexation occurred. The physical mixture of BR and β-CD showed a thermal event near 310 °C triggered by BR decomposition, and another thermal event near 330 °C caused by water decomposition from β-CD as revealed by TGA analysis. These results further confirmed that the BR molecule was encapsulated in the cavities of the β-CD after complexation.

Finally, this work evaluated the stability of BR/β-CD. BR was extremely unstable in solution. Hence, it was meaningful to evaluate the stability of BR/β-CD by measuring BR content exposed to sunlight. A similar volume of BR solution and BR/β-CD solution (with equal BR concentration) was placed in the bottle and recorded the appearance and UV absorption spectra within 7 days (Figure 1(G–J)). Moreover, the BR concentration was measured at specific time intervals (Figure 1(F)). Its concentration in solution was significantly decreased at day 3 and day 7, whereas that of BR/β-CD only slightly changed. Figure 1(G) shows that BR in the solution was quickly oxidized and the colour of BR solution turned to totally dark green after standing for 7 days. This was consistent with findings of the UV spectra. In contrast, BR/β-CD remained stable, and the solution colour remained unchanged after standing for 7 days (Figure 1(I)). Quantitative analysis verified the high BR concentration (Figure 1(F,J)). These results revealed that BR/β-CD had higher stability compared to BR.

### Characterization of bioadhesive SGP hydrogel containing BR/β-CD

Further, BR/β-CD/SGP hydrogel was prepared by mixing BR/β-CD with SGP hydrogel, and the physicochemical properties of BR/β-CD/SGP hydrogel were investigated by SEM, degradation testing, rheological testing, *in vitro* drug release, and biocompatibility. As shown in Figure 2(A), BR/β-CD was presented in a solution state. After compositing into SGP hydrogel, the prepared BR/β-CD/SGP hydrogel showed yellow colour with gel state. SEM was used to analyse the morphology of the BR/β-CD/SGP hydrogel. As shown in Figure 2(B), both SGP and BR/β-CD/SGP hydrogel displayed uniform structures with macro-porous, and the pore sizes of hydrogel networks ranged between 10 and 30 μm. The porous structure preserved moisture and oxygen exchange, hence promoted wound healing.

**Figure 2.** Characterization of BR/β-CD/SGP hydrogel. (A) The appearance of BR/β-CD solution, SGP, and BR/β-CD/SGP. (B) SEM images showed a cross-sectional morphology of SGP and BR/β-CD/SGP. (C) *In vitro* enzyme degradation rate of BR/β-CD/SGP. (D) Rheological behaviour of BR/β-CD/SGP. (E) Adhesive stress of different hydrogels. *In vitro* release profile of BR, BR/β-CD, and BR/β-CD/SGP in the (F) absence or (G) presence of H_2_O_2_. (H) Biocompatibility of BR/β-CD/SGP hydrogel. **p < 0.05 compared to control group; ^&&^*p* < 0.05 compared to BR solution group. Each group was paralleled three times.

The SGP hydrogel was used as a medical dressing for wound closures, and a controlled release matrix for therapeutics. Thus, non-ideal hydrogel degradation might cause compromised efficacy in wound healing. The degradation rate was evaluated by examining the weight loss in PBS solution with papain, and more than 50% of BR/β-CD/SGP hydrogel remained after 48 h (Figure 2(C)). The suitable stability met the period process of diabetic wound healing.

The rheological properties of BR/β-CD/SGP hydrogel was investigated by monitoring storage modulus (G′) and loss modulus (Gʺ) as angular frequency changes. The SGP hydrogel was developed by mixing the thiolated γ-PGA and poloxamer F127. As depicted in the Figure 2(D), Gʺ values of SGP hydrogel exceeded the G′ values in the range of 0.1–100 rad/s angular, indicating that SGP maintained a stable internal structure even under large deformation and presented as a solid-like form. Meanwhile, the Gʺ values were nearly parallel to the G′ values in SGP rheological behaviour, indicating a liquid-like state. Besides, the composition of BR/β-CD displayed a negligible effect on the rheological properties of SGP hydrogel. This phenomenon indicated a satisfactory elastic property and stable physical structure of BR/β-CD/SGP hydrogel.

The bioadhesive force, expressed as the detachment stress in dyne/cm^2^, was established from the minimal weights needed to detach the hydrogel from the surface of rat skin (Figure 2(E)). For comparison, the pure poloxamer F127 hydrogel (P) and non-thiolated γ-PGA and poloxamer F127 hydrogel (GP) at similar concentrations were used as a control. The addition of γ-PGA slightly increased the adhesive force potentially due to the hydrophilic residues capable of binding glycoproteins in γ-PGA. More importantly, thiolated γ-PGA significantly enhanced bioadhesivity as evidenced by the significantly increased adhesive force. Moreover, the composition of BR/β-CD did not affect the bioadhesivity. These results indicated that thiolated γ-PGA contributed to the excellent bioadhesivity of SGP hydrogel.

The *in vitro* release behaviour of BR from the BR/β-CD/SGP hydrogel was further investigated. As shown in Figure 2(F), significantly limited BR was released into the dissolution medium due to the extremely low solubility in the pH 7.4 PBS solution. After inclusion complexation, the aqueous solubility of BR was significantly increased. Therefore, over 65% BR could be released from the BR/β-CD inclusion complex after 96 h. After loading into the hydrogel matrix, BR/β-CD/SGP hydrogel exhibited sustained BR behaviour and a slower release rate. Furthermore, we investigated the release profile of BR/β-CD/SGP hydrogel in the PBS with 10 mM H_2_O_2_ for stimulating the abundant ROS environment in the diabetic wound (Figure 2(G)). As expected, BR was released at a faster rate under H_2_O_2_ due to the higher solubility in a ROS abundant medium (Yao, Chen, et al. 2020). BR/β-CD complex inclusion enormously increased BR release rate, representing elevated solubility. Besides, it was noted that the BR release ratio from BR/β-CD/SGP hydrogel increased to nearly 40% in 48 h, significantly exceeding that in the PBS without H_2_O_2_, which was attributed to the redox reaction of sulfhydryl.

Since cytocompatibility is an important property that determined the medical application of biomaterials, HUVEC was co-cultured with BR/β-CD/SGP hydrogel in a series of BR concentration (10, 20, 30, 40, 50, 60 μM) for 24 h. The cell viability was assessed using the MTT assay (Figure 2(H)). BR at a higher concentration (>50 μM) induced a slight cytotoxic effect on the endothelial cells, which is consistent with our previous findings (Yao, Jiang, Huang, et al. 2019; Yao, Huang, et al. 2020). Nonetheless, 50 μM and even 60 μM equivalent BR/β-CD/SGP hydrogel did not impact the cell viability, and the viability of treated cells remained higher than 95%. No significant difference was observed between BR/β-CD inclusion complex and BR/β-CD/SGP hydrogel, which could be explained by the sustained release of BR from the inclusion complex and hydrogel system (Figure 2(F,G)), thus preventing sudden exposure of high concentration of BR.

These results demonstrated that BR/β-CD/SGP hydrogel had favourable elastic property, applicable stability, efficient biocompatibility, and redox responsive performance suitable for diabetic wound therapy.

### BR/β-CD/SGP accelerated cell proliferation and migration *in vitro*

Endothelial cell proliferation and migration played a pivotal role in the angiogenesis and tissue remodelling which were in disorder in the diabetic wound healing (Du et al. 2018). Therefore, the effect of BR/β-CD/SGP hydrogel on HUVEC proliferation and migration rate was investigated using an *in vitro* scratch test. The wounds were photographed at 0 and 24 h post-scraping. As shown in Figure 3, different drug treatments caused a significant difference in wound closure and cell viability. Blank processing induced a delayed wound closure, and BR/β-CD/SGP hydrogel significantly increased the wound close area compared to blank treatment (*p* < 0.05) and BR treatment (*p* < 0.05), indicating that BR/β-CD/SGP hydrogel markedly improved cell migratory rate (Figure 3(A,B)). The cell proliferation rate of the BR/β-CD/SGP group was significantly higher compared to the control group (*p* < 0.05) and BR group (*p* < 0.05), further verifying the protecting effect of the BR/β-CD/SGP hydrogel on the endothelial cells (Figure 3(C)). These results demonstrated that BR/β-CD/SGP hydrogel accelerated *in vitro* cell proliferation and migration.

**Figure 3.** Cell migration and proliferation of HUVEC cells with treatments of BR, BR/β-CD, BR/β-CD/SGP hydrogel. (A) The images of HUVEC cell migration were recorded at 0 h (above) and 24 h (below) after scraping. Magnification: 100×. (B) The calculated wound closure rate. (C) The effect of BR, BR/β-CD, BR/β-CD/SGP on HUVEC proliferation was investigated using MTT assay. Data are shown as mean ± SD (*n* = 3). **p < 0.05 compared to control group; ^&&^*p* < 0.05 compared to the BR solution group.

### BR/β-CD/SGP promoted the diabetic wound healing *in vivo*

To investigate the pro-healing efficiency of BR/β-CD/SGP, BR solution or BR/β-CD/SGP was applied on diabetic rats post-wound surgery. Normal rats post-wound surgery was administered with or without BR/β-CD/SGP. As depicted in Figure 4(A), the wounds of each group were photographed on day 3, 7, 14, and 21 after wound surgery. All the groups appeared to contract wound with time but demonstrated different healing rate. Based on previous studies, it was observed that diabetic wounds without treatment had the slowest rate of healing (Sambasevam et al. 2013; Ahanger et al. 2016). BR solution treatment significantly elevated the diabetic wound closure at day 7 (*p* < 0.05) and day 14 (*p* < 0.05) (Figure 4(B)). Moreover, normal rats or diabetic rats post wound surgery treated with BR/β-CD/SGP significantly increased the wound closure at day 3 (*p* < 0.05), day 7 (*p* < 0.05), and day 14 (*p* < 0.05), indicating an improved healing property of BR/β-CD/SGP. By comparison, BR/β-CD/SGP treatment showed higher pro-healing efficiency than BR solution, which was explained by the better bioavailability and addressing advantage of BR/β-CD/SGP. Further, H&E staining was performed to observe the pathology condition (Figure 4(C)). The skin tissue at day 3 after surgery was significantly slim and thin with no formed neo-epidermis, while the skin tissue at day 7 appeared thick in the granulation tissue with the reduction of wound length, even recovered hair follicle tissue at the injured sites. Results of the quantitative analysis of wound length at day 3 (Figure 4(D)) and day 7 (Figure 4(E)) were consistent with the aforementioned findings. The length of the diabetic wound was longest at day 3 and day 7. Besides, BR/β-CD/SGP treatment significantly reduced wound length in both normal and diabetic rats post-wound surgery (*p* < 0.05). Although the BR solution reduced the length of diabetic wounds, the reduction was less than that of the BR/β-CD/SGP treatment (*p* < 0.05). In addition, we found that BR/β-CD/SGP promoted diabetic wound healing more efficiently compared to BR solution.

**Figure 4.** BR/β-CD/SGP hydrogel accelerated wound closure. (A) Representative images of wound healing process treated with BR or BR/β-CD/SGP hydrogel on both normal (Nor) or diabetic rats (DM). (B) Wound closure of all five groups. (C) H&E staining images of full-thickness wounds on days 3 and 7; arrows indicate the centre of the wound, scale bar: 500 μm. Quantification of the wound length at (D) day 3 and (E) day 7. Data are shown as mean ± SD (*n* = 6). **p < 0.05 compared to DM control group; ^^*p* < 0.05 compared to normal control group; ^@@^*p* < 0.05 compared with BR-treated DM group.

### BR/β-CD/SGP promoted diabetic wound healing by inhibiting inflammation

Macrophages function as scavengers that remove apoptotic neutrophils and wound debris. They also initiate inflammation during wound healing. The polarization of macrophages from M2 to M1 promotes inflammation reaction leading to the release of inflammatory cytokines. The skin tissue was collected at day 3 post-wound injury to analyze macrophage and neutrophils infiltration by immunohistochemistry. CD86 and MPO were selected as markers of macrophages-1 (M1) and neutrophils, respectively (Li et al. 2020). As shown in Figure 5(A), the diabetic wound had large areas of CD86-positive staining and MPO-positive staining, indicating high macrophage and neutrophil infiltration. This phenomenon was observed in normal wounds. By contrast, BR/β-CD/SGP treatment significantly decreased the CD86-positive area (∼67%) and MPO-positive area (∼77%) in diabetic wound, indicating that the infiltration level of macrophage and neutrophils was suppressed. BR/β-CD/SGP treatment in normal wounds also showed good outcomes. Treatment with BR effectively reduced macrophage and neutrophil infiltration, but not as strong as BR/β-CD/SGP (*p* < 0.05). These results were further verified by quantitative analysis (Figure 5(B,C)). The interaction between inflammatory cytokines and inflammatory cell infiltration suppressed wound healing. Therefore, the TNF-α expression was further investigated in these skin tissue (Figure 5(A)). TNF-α showed a similar tendency with CD86 and MPO, manifested by the larger TNF-α-positive area in the DM group compared to those in the DM-BR (*p* < 0.05) and DM-BR/β-CD/SGP (*p* < 0.05) groups (Figure 5(D)). A high level of TNF-α was confirmed to strongly impact wound healing, including the inhibition of fibroblast migration and endothelial progenitor cells (EPC) mobilization, remarkably, stimulating the polarization of the macrophage (Snyder et al. 2016). Combined with the aforementioned wound repair situation on day 3, this case was interpreted as that of inflammatory cell maliciously and excessively recruited in the wound healing. BR/β-CD/SGP treatment also deceased TNF-α expression in wounds of normal rats. These data indicated that BR/β-CD/SGP promoted diabetic wound healing by inhibiting both inflammatory cytokines and inflammatory cell infiltration.

**Figure 5.** (A) Immunohistochemical analysis of CD86, MPO, and TNF-α at day 3 post wound injury. Scale bar: 100 μM. The corresponding quantitative analysis of (B) CD86, (C) MPO, and (D) TNF-α. Data are presented as mean ± SD (n = 3). ^^, p < 0.05 compared to normal wound group; **, p < 0.05 compared to diabetic wound group; @@, p < 0.05 compared to BR-treated diabetic wounds.

### BR/β-CD/SGP accelerates diabetic wound healing by promoting collagen deposition and upregulating FGF-1 and VEGF

The climax of inflammation overlapped with the proliferative phase during the wound healing process. This stage was characterized by fibroblast migration, endothelial cell proliferation, causing collagen deposition and neovascularity (Shah et al. 2019). Collagen deposition influences the wound healing process. Collagen IV is a crucial component of the extracellular matrix (ECM) present in the extracellular basement membranes separating the epithelial cells and endothelial cells. The expression of collagen IV was examined by immunohistochemistry on day 7 after wound injury to assess this process (Figure 6(A)). The diabetic wound exhibited a lower collagen IV positive area than the normal wound, which was diminutively elevated to almost 35% by BR treatment (*p* < 0.05), but more strongly elevated up to 80% by BR/β-CD/SGP treatment (*p* < 0.05) (Figure 6(B)). BR/β-CD/SGP treatment upregulated collagen IV expression in normal wounds. TGF-β played a favourable role in the fibroblast migration and keratinocyte migration, resulting in accelerated re-epithelialization and collagen deposition (Guo et al. 2020). Diabetic wound and normal wound all exhibited few TGF-β-positive areas, slightly elevated by BR treatment (*p* < 0.05), but significantly increased to 60% by BR/β-CD/SGP treatment (*p* < 0.05) (Figure 6(C)). Fibronectin played a vital role in all stages of wound repair, and fibronectin promoted fibroblasts migration and deposit with the collagen-III in interstitial cells in the middle of the wound repair (Lenselink 2015). The fibronectin positive area was scarcely detected in the diabetic wound, comparably increased in normal wound (Figure 6(D)). Both BR and BR/β-CD/SGP treatment significantly increased the fibronectin positive areas; with the latter producing a more pronounced increase (*p* < 0.05). These results indicated that BR/β-CD/SGP effectively elevated collagen-IV, TGF-β, and fibronectin levels in diabetic wounds, hence promoting collagen deposition.

**Figure 6.** (A) Immunohistochemical analysis of Collage IV, TGF-β, FN, VEGF, FGF-1 at day 14 post wound injury. Scale bar: 100 μM. The corresponding quantitative analysis of (B) Collage IV, (C) TGF-β, (D) FN, (E) VEGF, and (F) FGF-1. Data are presented as mean ± SD (*n* = 3). ^^*p* < 0.05 compared to the normal wound group; **p < 0.05 compared to diabetic wound group; ^@@^*p* < 0.05 compared to BR-treated diabetic wounds.

Microcirculatory disturbances delay the healing process of diabetic wounds. In angiogenesis, VEGF regulates revascularization at the wound site (Shao et al. 2019). VEGF increased the capillary density hence blood perfusion in diabetic wound tissue, which promotes the healing process. The VEGF expression was established to evaluate the therapeutic effect of BR/β-CD/SGP. As shown in Figure 6(A,E), diabetic wounds exhibited little VEGF-positive area, fewer than normal area. BR/β-CD/SGP remarkably elevated VEGF-positive area in both normal (*p* < 0.05) and diabetic (*p* < 0.05) wounds, the efficacy of which was higher than BR treatment (*p* < 0.05). It was reported that FGF-1 stimulated mitosis and migration of vascular endothelial cells, epidermal keratinocytes, and dermal fibroblasts (Blaber et al. 2015). In the present study, BR/β-CD/SGP and BR upregulated the expression of FGF-1 in both normal and diabetic wounds, and BR/β-CD/SGP showed significantly better performance compared to BR (Figure 6(F)). The superior performance of BR/β-CD/SGP was probably attributed to its good sustained BR release profile and bioavailability. These results demonstrated that BR/β-CD/SGP potentially promotes diabetic wound healing by upregulating VEGF and FGF-1.

## Conclusions

This work designed and characterized a bioadhesive hydrogel (BR/β-CD/SGP) containing bilirubin/β-cyclodextrin inclusion complexes for diabetic wound treatment. The bioadhesive property of hydrogel kept the drug-containing hydrogel attached to the wound tissue, thereby enhancing the recovery of skin appearance and texture. The prepared BR/β-CD/SGP exhibited a sustained release profile of BR, hence triggered strong anti-inflammatory effects to promote tissue remodelling during diabetic wound healing process. These findings demonstrated that BR/β-CD/SGP hydrogel can be used to promote wound healing and treat inflammatory diseases.
